This article has been retracted.

# Giant Unruptured Internal Carotid Artery Aneurysm

**DOI:** 10.7759/cureus.20423

**Published:** 2021-12-15

**Authors:** Sultan O Gohal, Abrar A Alally, Abdulaziz I Alhonaizil, Abdulelah A Alabdulwahab, Khalid S Alzahrany, Mohammed A Alomari, Faisal A Alshunaibir, Mohammed A Alsalman, Naif M Alhamyani, Hamzah M Alamri, Ali A Alharbi, Abdulmohsen J Alabood, Fahad S Alshahrani, Adam M Al Amer, Faisal Al-Hawaj

**Affiliations:** 1 College of Medicine, Batterjee Medical College, Jeddah, SAU; 2 Faculty of Health, Medicine and Life Sciences, Maastricht University, Maastricht, NLD; 3 College of Medicine, AlMaarefa University, Ad Diriyah, SAU; 4 College of Medicine, King Faisal University, Hofuf, SAU; 5 College of Medicine, Medical University of Lodz, Lodz, POL; 6 College of Medicine, King Abdulaziz University, Jeddah, SAU; 7 College of Medicine, Imam Abdulrahman Bin Faisal University, Dammam, SAU; 8 College of Medicine, Al-Baha University, Al-Baha, SAU; 9 College of Medicine, Qassim University, Qassim, SAU; 10 College of Medicine, Vision Colleges, Riyadh, SAU; 11 College of Medicine, King Khalid University, Abha, SAU

**Keywords:** case report, surgical clipping, internal carotid artery, aneurysm, headache

## Abstract

Headache is among the most frequent symptoms to seek medical care. Careful evaluation by history-taking and appropriate physical examination is needed to exclude the potential secondary causes of headaches. In the elderly population, secondary headaches are more prevalent compared with the younger adult population. We present the case of a 70-year-old man who presented with a three-month history of headache with visual disturbances. He reported that this was the first time he experienced such a headache. The patient had a longstanding history of hypertension, diabetes mellitus, dyslipidemia, and ischemic heart disease. He was a heavy smoker with a 35 pack-years smoking history. In view of the clinical signs and symptoms, the patient underwent a computed tomography scan that revealed a right internal carotid artery aneurysm. For better evaluation, magnetic resonance imaging of the brain was performed and re-demonstrated the saccular aneurysm of the terminal part of the right internal carotid artery aneurysm, measuring 48 x 37 x 31 mm and partially thrombosed with a surrounding mural hematoma. The neck of the aneurysm measured 4 mm. The decision for surgical management was planned. The patient underwent craniotomy with surgical clipping of the aneurysm. No complications occurred during the operation. The patient had an uneventful recovery. Elderly patients with chronic headaches should be carefully evaluated for secondary headaches. A giant cerebral artery aneurysm is an uncommon etiology of secondary headache that needs prompt diagnosis and management.

## Introduction

Headache is the most common neurologic complaint and is among the most frequent reasons to visit the emergency department. It affects over 50% of the population at any point in time [1]. However, the prevalence of headaches decreases with age. The etiology of headaches can be divided into primary and secondary headaches. In the elderly, the primary headache is twice more common than the headache due to secondary causes [2]. However, elderly patients should be carefully evaluated for the possibility of secondary etiologies for their headaches. A prior study showed that the elderly populations are more than 10 times likely to have secondary headaches compared with the adult population [3]. Therefore, a comprehensive assessment with complete history taking and neurological examination are crucial. Laboratory and imaging studies are indicated if there were any “red flags.” Computed tomography is often the first-line imaging modality for the assessment of acute headaches. Further, magnetic resonance imaging is indicated for chronic headaches. The secondary etiologies of headache include giant cell arteritis, intracranial malignancy, ischemic strokes, glaucoma, subarachnoid and subdural hematoma, and meningitis [1]. Here, we present the case of an elderly patient with chronic headache and visual deficit who was eventually diagnosed as having a giant unruptured internal carotid artery aneurysm.

## Case presentation

We present the case of a 70-year-old man who was brought to the emergency department by his son because of a three-month history of headaches. He reported that the headache was generalized and described it as having a pressure-like quality. It was non-radiating. He first noted it for three months, and it had been increasing in severity. It was constant and partially relieved by non-steroidal anti-inflammatory drugs. It was not disturbing his sleep. There was no history of fever, nausea, or vomiting with the headache. However, the patient reported a decline in his visual impairment in both eyes. He reported that this was the first time him to experience such a headache. He scored it as 7 out of 10 on the severity scale.

Regarding past medical history, the patient had a longstanding history of hypertension, diabetes mellitus, dyslipidemia, and ischemic heart disease. His conditions were under good control. He was on aspirin 75 mg, captopril 5 mg, atorvastatin 20 mg, and metformin 1 g for the management of his comorbid conditions. His surgical histories included open cholecystectomy and appendectomy. He was a heavy smoker with a 35 pack-years smoking history but he never consumed alcohol. He was a retired electrical engineer, and his family history was unremarkable.

Upon examination, the patient appeared drowsy and tired. He was oriented to time, place, and person. Examination of the higher mental status function was normal. Cranial nerves examination showed decreased visual fields bilaterally with decreased visual acuity. Otherwise, there were no signs of focal neurological deficits. Both the upper and lower extremities had a normal tone and power. Coordination was intact, with normal knee and ankle reflexes. The Babinski sign was negative.

Initial laboratory investigation showed normal results. The hematological findings revealed a hemoglobin level of 14.2 g/dL, leukocyte count of 8200/μL, and platelet count of 388,000/μL. The inflammatory markers, including erythrocyte sedimentation rate (14 mm/hr.) and C-reactive protein (5.1 mg/dL), were within the normal rates. Renal function tests revealed normal levels of blood urea nitrogen (12 mg/dL), creatinine (1.2 mg/dL), and electrolytes. The liver enzymes were not elevated (Table 1).

**Table 1:** Summary of the results of laboratory findings

Laboratory Investigation	Unit	Result	Reference Range
Hemoglobin	g/dL	14.2	13.0–18.0
White Blood Cell	1000/mL	8200	4.0–11.0
Platelet	1000/mL	388	140–450
Erythrocyte Sedimentation Rate	mm/hr.	14	0–20
C-Reactive Protein	mg/dL	5.1	0.3–10.0
Total Bilirubin	mg/dL	0.9	0.2–1.2
Albumin	g/dL	3.9	3.4–5.0
Alkaline Phosphatase	U/L	52	46–116
Gamma-Glutamyltransferase	U/L	17	15–85
Alanine Transferase	U/L	18	14–63
Aspartate Transferase	U/L	20	15–37
Blood Urea Nitrogen	mg/dL	12	7–18
Creatinine	mg/dL	1.2	0.7–1.3
Sodium	mEq/L	137	136–145
Potassium	mEq/L	3.9	3.5–5.1
Chloride	mEq/L	104	98–107

In view of the clinical signs and symptoms, the patient underwent a computed tomography scan with intravenous contrast to rule out any space-occupying lesion. The scan revealed a right internal carotid artery aneurysm (Figure 1). For better evaluation, magnetic resonance imaging of the brain was performed. The scan demonstrated a saccular aneurysm of the terminal part of the right internal carotid artery aneurysm, measuring 48 x 37 x 31 mm, which was partially thrombosed with a surrounding mural hematoma. The neck of the aneurysm measured 4 mm. The aneurysm had no arterial branches arising from it and was exerting a pressure effect on the optic chiasm and the lateral ventricles. Such findings conferred the diagnosis of a giant internal carotid artery aneurysm (Figure 2).

**Figure 1:** Coronal CT head angiography demonstrates a large saccular aneurysm (arrow) of the right internal carotid artery. CT: computed tomography

**Figure 2:** Axial (A) and sagittal (B) MR T2-weighted images demonstrate a partially thrombosed giant internal carotid artery aneurysm MR: magnetic resonance

Considering the giant size of the aneurysm and the wide neck, the decision for surgical management was planned. The option was discussed with the patient and high-risk consent was taken. The patient underwent craniotomy with surgical clipping of the aneurysm. No complications occurred during the operation. The patient had an uneventful recovery. No signs of ischemia were noted and the patient was discharged after 10 days of hospitalization. After three months of follow-up, the patient remained asymptomatic.

## Discussion

We presented the case of a giant unruptured internal carotid artery aneurysm that presented with chronic headache and visual impairment. A giant cerebral artery is defined as having a maximum dimension of greater than 25 mm [4]. Only 5% of intracranial aneurysms have such size. The risk of rupture of giant cerebral artery aneurysms is 6% per year [4]. Notably, it is reported that over 50% of giant cerebral arteries present with rupture [5].

The pathogenesis of giant cerebral aneurysm includes de novo development as a result of weakness in the elastic lamina of the vessel or it may develop after progression of a smaller aneurysm due to turbulent flow and hemodynamic stress [5]. As in the present case, the vast majority of intracranial aneurysms have a saccular type. In contrast, fusiform aneurysms include a longer segment of the artery and are often developed in patients with extensive atherosclerosis [4].

Several risk factors have been described as associated with giant cerebral aneurysms. These factors include typically advanced age, smoking, and hypertension. In our patient, all of these factors were present [6]. In addition, a cerebral aneurysm is more prevalent among female patients. Certain connective tissue disorders, including Marfan syndrome, adult polycystic kidney disease, and Ehler-Danlos syndrome, are known associations with intracranial aneurysms [4]. It is crucial to note that the factors that predispose to the formation of intracranial aneurysms are themselves the factors that increase the risk for aneurysmal rupture [5].

The clinical manifestation of cerebral artery aneurysms primarily depends on their size and location [5]. Ruptured aneurysm causing subarachnoid hemorrhage classically present with severe thunderclap headache that may be associated with loss of consciousness. In contrast, an unruptured aneurysm typically presents with signs and symptoms of the space-occupying lesion [4]. In our case, the patient presented with chronic headache and bitemporal hemianopia because of the suprasellar location of the aneurysm causing compression on the optic chiasm. In addition, the unruptured aneurysm can have a wide range of presentations, including cranial nerve palsies, seizures, and ischemic strokes due to thromboembolism [6].

Cross-sectional studies can make the diagnosis of giant cerebral artery aneurysms with high accuracy. Further, the use of computed tomography or magnetic resonance imaging angiography is of paramount importance for better characterization and assessment of the aneurysm in terms of its flow, anatomic relationship, and the aneurysm neck [6]. The management of a giant cerebral aneurysm is challenging. It depends highly on the aneurysm size, aneurysm type, neck size, presence of collateral circulation, and other factors [4]. In the present case, surgical clipping was performed because of the wide neck and large size of the aneurysm causing a pressure effect.

## Conclusions

Elderly patients with chronic headaches should be carefully evaluated for secondary headaches. A giant cerebral artery aneurysm is an uncommon etiology of secondary headache that needs prompt diagnosis and management. The diagnosis can be established by cross-sectional studies with angiography. Early management can be life-saving to avoid the catastrophic outcome of ruptured aneurysms.
